The article "Relationship between the Autoantibody and Expression of β3-Adrenoceptor in Lung and Heart" was retracted in 2025. Reasons: errors in the images; duplicated images; overlap with earlier publications; unreliable results or conclusions.

# Relationship between the Autoantibody and Expression of β_3_-Adrenoceptor in Lung and Heart

**DOI:** 10.1371/journal.pone.0068747

**Published:** 2013-07-05

**Authors:** Guobin Miao, Zhe Chen, Xiangyang Fang, Miaobing Liu, Gang Hao, Huiling An, Zhiyong Zhang, Lingqiao Lu, Jian Zhang, Lin Zhang

**Affiliations:** 1 Department of Internal Medicine, Beijing Chaoyang Hospital, Capital Medical University, Beijing, China; 2 Department of Pathophysiology, Capital Medical University, Beijing, China; 3 Heart Failure Center, Department of Cardiology, Beijing Chaoyang Hospital, Capital Medical University, Beijing, China; 4 Medical and Health Center, Beijing Friendship Hospital, Capital Medical University, Beijing, China; Cardiovascular Research Institute Maastricht, Maastricht University, The Netherlands

## Abstract

**Background:**

Evidences suggest that β_3_ **-**adrenoceptor (β_3_-AR) plays an important role in heart failure (HF), although no data is reported indicating how these effects may change with the increasing age. Pulmonary congestion and edema are the major life-threatening complications associated with HF. The purpose of this study is to explore the relationship between the anti-β_3_-AR autoantibody and the expression of β_3_-AR in the lungs and heart for both aged patients and rats with HF.

**Methods:**

Synthetic β_3_-AR peptides served as the target antigens in ELISA were used to screen the anti-β_3_-AR autoantibody in aged patients and rats. Two aged rat models were constructed based on aortic banding and sham-operation. The expression of β_3_-AR mRNA and protein in the lung and heart was measured in intervention and non-intervention groups by Western blot analysis at the baseline, 5^th^, 7^th^, 9^th^ and 11^th^ week, respectively.

**Results:**

The frequency and titer of anti-β_3_-AR autoantibody in aged patients and rats with HF were higher than those in the control group (*p*<0.05). The expression of β_3_-AR mRNA and protein in pulmonary tissues decreased continually from the 7^th^ week (*p*<0.05), followed by HF observed during the 9^th^ week. The expression of β_3_-AR in myocardial tissues continued to increase after the 9^th^ week (*p*<0.05), and the expression of both β_3_-AR mRNA and protein in the BRL group [HF group with BRL37344 (4-[-[2-hydroxy-(3-chlorophenyl)ethyl-amino] phenoxyacetic acid) (a β_3_-AR agonist) injection] was positively correlated with BRL37344 when compared with non-BRL group (HF group without BRL37344 injection) (*p*<0.05).

**Conclusion:**

Anti-β_3_-AR autoantibody was detected in aged patients and rats with HF. The expression of β_3_-AR mRNA and protein in pulmonary tissues decreased continually, and began earlier than in the heart, but its expression in myocardial tissues increased continually and could be further promoted by β_3_-AR agonist.

The article "Relationship between the Autoantibody and Expression of β3-Adrenoceptor in Lung and Heart" was retracted in 2025. Reasons: errors in the images; duplicated images; overlap with earlier publications; unreliable results or conclusions.

## Introduction

Growing evidences suggest that the autoimmune mechanism may play a major role in heart failure observed in both rats and human patients [1], [2], [3], [4]. Previous studies have shown that autoantibodies against β-adrenoceptors (anti-β-AR autoantibodies) display antagonist activity on the corresponding receptor and influence cardiac function [3], [5], [6] It has been well established that β-adrenoceptor (β-AR) belongs to the family of G-protein coupled receptors, and 3 subtypes (β_1_, β_2_ and β_3_-AR) have been associated with different changes in heart failure. Stimulation to β_1_ and β_2_-AR produces positive chronoscopic and inotropic effects. However, the activation of β_3_-AR induces a decrease in the contractility of myocardium [7], [8], [9], [10]. Gauthier and associates recently have also reported that β_3_-AR is obviously coupled to a Gi/nitric oxide (NO) pathway and can reveal negative inotropic effects in ventricular endomyocardial biopsy samples of heart transplant recipients [11]. However, some disagreement exists regarding the conclusions reported by these studies [8], [12], thus indicating that the relationship between β_3_-AR and cardiac function warrants further investigation, in aged patients or rats with heart failure.

Pulmonary congestion and edema are the major life-threatening complications associated with heart failure. The β-AR is widely distributed in lungs, where the dominant subtype is β_2_-AR [13]. Recently, the research has found that the administration of an inhaled β_2_-AR agonist can improve pulmonary function in patients with congestive heart failure, thus suggesting the involvement of β_2_-AR [14]. Other studies have found that β_2_-agonist can increase alveolar fluid clearance in rats with heart failure [15]; however, the other 2 subtypes (β_1_-AR and β_3_-AR) in pulmonary tissues have gained less attention. Recent research has demonstrated very low expression of β_3_-AR mRNA in the lungs, and the authors have suggested that the expression of β_3_-AR mRNA could probably be accounted for by the presence of fat [16]. Additionally, new research has confirmed the presence of β_3_-ARs in human bronchi [13], and has further indicated that β_3_-adrenergic agonists may also increase alveolar fluid clearance during hypoxic lung injury in rats, and accelerate the amelioration of pulmonary edema [17].

The major objectives of this study are summarized by three hypotheses: 1) The anti-β_3_-AR autoantibodies can be detected in the plasma of aged patients and rats with heart failure. 2) The abnormal expressions of β_3_-AR mRNA and protein, and changes in the levels of anti-β_3_-AR autoantibodies in pulmonary congestion or edema emerge prior to the appearance of heart failure in aged rats. 3) These latter changes may involve continuing deterioration during heart failure, and may further be altered by the introduction of the β_3_-AR agonist.

The article "Relationship between the Autoantibody and Expression of β3-Adrenoceptor in Lung and Heart" was retracted in 2025. Reasons: errors in the images; duplicated images; overlap with earlier publications; unreliable results or conclusions.

## Results

### Mortality Rate of Aged Rats

Mortality rate with Banded group was significantly higher than that in the Sham group (*p*<0.01, 50.0% *vs.* 8.6%) during the postoperative period (0–11 weeks). The major causes of early death were over anesthesia or heart failure, especially in the Banded group. From the 5^th^ week, the rats from the Banded group (n = 90) were divided randomly into two groups as the BRL group [heart failure group with a β_3_-AR agonist called BRL37344 (4-[-[2-hydroxy-(3-chlorophenyl)ethyl-amino] phenoxyacetic acid) injection] (n = 50) and the non-BRL group (heart failure group without BRL37344 injection) (n = 40). Mortality rates were different at various stages in the non-Banded and BRL groups from the 5^th^ to 11^th^ week. The accumulative mortality rate in the BRL group was significantly higher than that in the non-BRL group (*p*<0.05, 32% *vs.* 12%), and these results suggested that β_3_-AR agonist (BRL37344) might be associated with an increased risk of death in aged rats with heart failure.

### Hemodynamic Parameters and Left Ventricle/Body Weight Ratio

The hemodynamic parameters are summarized in Table 1. In both the BRL group and the non-BRL group, the HR, LVESP and dP/dt_max_ decreased, and LVEDP and dP/dt_min_ increased significantly, when compared with the Sham group (*p*<0.05). However, at the 9^th^ week, left ventricular function was significantly impaired in the BRL group compared to the non-BRL group (*p*<0.01). Thus, left ventricular function was progressively damaged.

**Table 1:** Hemodynamic effects following injection.

Group	Time	N	HR	LVESP	LVEDP	dp/dt max	dp/dt min
	(Weeks)		(bpm)	(mm Hg)	(mm Hg)	(mmHg/ms)	(mmHg/ms)
Sham	5	8	353±27	154.9±12.5	0.96±0.60	9.40±0.97	–6.28±0.52
	7	8	379±15	154.1±3.0	1.01±0.53	9.38±0.50	–6.08±0.35
	9	8	395±15	152.6±4.0	0.90±0.40	9.08±0.52	–5.80±0.62
	11	8	394±16	153.8±5.2	0.89±0.49	9.38±0.26	–6.08±0.54
Non-BRL	5	8	364±29	178.3±6.1*	7.25±0.71*	8.88±1.87	–6.29±0.76
	7	8	381±32	173.2±9.3*	7.47±0.76*	8.74±1.56	–5.72±0.95
	9	8	269±20*	88.3±7.5*	10.31±1.62*	5.85±0.76*	–2.68±0.55*
	11	8	254±14*	61.5±2.4*	10.74±0.48*	1.40±0.21*	–1.18±0.41*
BRL	5	8	356±11	178.3±1.8*	7.30±0.98*	9.94±1.66	–6.50±0.78
	7	8	370±13	170.9±7.6*	7.69±0.83*	8.35±0.51	–5.81±0.17
	9	8	222±23* ‡	73.2±7.8* ‡	11.13±0.61*	2.36±1.19* ‡	–1.84±0.75*
	11	8	216±20* ‡	42.5±3.8* ‡	12.17±0.50* ‡	1.75±0.52*	–1.08±0.33*

Data are presented as means ± standard error. Sham: control group; Non-BRL: HF group without BRL37344 injection; BRL: HF group with BRL37344 injection; HR: heart rate; LVESP: left ventricular end-systolic pressure; LVEDP: left ventricular end-diastolic pressure; dp/dt max: maximum rate of rise of left ventricular pressure; dp/dt min: maximum rate of fall of left ventricular pressure.

* *P*<0.01 vs. Sham group;

† *P*<0.05 vs. Non-BRL group;

‡ *P*<0.01 vs. Non-BRL group.

The article "Relationship between the Autoantibody and Expression of β3-Adrenoceptor in Lung and Heart" was retracted in 2025. Reasons: errors in the images; duplicated images; overlap with earlier publications; unreliable results or conclusions.

The left ventricle weight and left ventricle weight/body weight ratio in both BRL group and non-BRL group were significantly higher than those in the Sham group, but overall body weight was lower. However, the average ratio in the BRL group was significantly higher than in the non-BRL group at the 7^th^ week (Table 2). Body weight did not reveal a significant difference between non-BRL and BRL groups. Our results indicate that left ventricular function was significantly reduced in the BRL group.

**Table 2:** The ratio of left ventricle weight to body weight following injection.

Group	Time (Weeks)	N	BW (g)	LVW (g)	LV/BW (mg/g)
Sham	5	8	529±13	1.00±0.04	1.89±0.06
	7	8	585±29	1.11±0.02	1.89±0.03
	9	8	601±19	1.09±0.07	1.81±0.10
	11	8	622±23	1.15±0.07	1.85±0.06
					
Non-BRL	5	8	485±29†	1.07±0.08†	2.22±0.18†
	7	8	574±36	1.28±0.09*	2.24±0.17†
	9	8	584±27	1.34±0.06†	2.30±0.11†
	11	8	581±16†	1.35±0.05†	2.32±0.09†
					
BRL	5	8	484±33†	1.06±0.13	2.19±0.29†
	7	8	595±35	1.45±0.21† ‡	2.42±0.22† ‡
	9	8	591±57	1.48±0.19† ‡	2.50±0.21† ‡
	11	8	596±26*	1.51±0.17† §	2.52±0.23† ‡

Data are presented as means ± standard errors. Sham: control group; Non-BRL: HF group without BRL37344 injection; BRL: HF group with BRL37344 injection; BW: body weight; LVW: left ventricular weight; LV/BW: left ventricular weight/body weight.

* *P*<0.05 vs. Sham group;

† *P*<0.01 vs. Sham group;

‡ *P*<0.05 vs. Non-BRL group;

§ *P*<0.01 vs. Non-BRL group.

### Anti-β_3_-AR Autoantibody in Aged Patients and Rats

The frequencies of anti-β_3_-AR autoantibody in aged patients with heart failure were 39.6% (mean antibody titer: 142.3±3.1), which was obviously higher than 12.7% (mean antibody titer: 64.3±3.1) in aged control group.

Similar results were observed in aged rats with heart failure. The frequencies and mean titer of anti-β_3_-AR autoantibody in the Banded group increased significantly from the 5^th^ week, with a high peak (from 20.4% and 28.3±1.4 to peak 41.4% and 82.3±3.2) at the 10^th^ week, followed by a decrease after the 10^th^ week, although these results were not observed in the Sham group (*p*<0.05). It was worth noting that the frequencies and mean titers of anti-β_3_-autoantibodies in the BRL group increased markedly at the 5^th^ week, and reached a maximum at the 10^th^ week (from 37.5% and 68.4±2.3 to peak 66.5% and 142.6±1.1) when compared with the Sham group (*p*<0.05) (Figure 1).

The article "Relationship between the Autoantibody and Expression of β3-Adrenoceptor in Lung and Heart" was retracted in 2025. Reasons: errors in the images; duplicated images; overlap with earlier publications; unreliable results or conclusions.

**Figure 1:** The frequencies of anti-β_3_-autoantibodies in non-BRL and BRL groups of aged rats with heart failure. 2 mL of blood samples were collected before treatment, and at the 5^th^, 6^th^,7^th^, 8^th^,9^th^, 10^th^ and 11^th^ week after treatment. The sera were separated by centrifugation (3000 rpm, Beckman CS-15R Centrifuge) for 10 min and stored at −80°C until needed for assay. Anti-β_3_-AR autoantibody was determined by enzyme-linked immunosorbent assays (ELISA). The frequencies of anti-β_3_-autoantibodies in the BRL group increased markedly at the 5^th^ week, and reached a maximum at the 10^th^ week in both BRL group and non-BRL group. The frequencies of anti-β_3_-autoantibodies were significantly higher in BRL group than non-BRL group and Sham group (*p<0.05). BRL group: HF group with β_3_-AR agonist of BRL37344 injection; non-BRL group: HF group without BRL37344 injection.

### Lung Histopathology in Aged Rats With Heart Failure

To our knowledge, this is the first reported observation of the changes occurring in the lungs (the 7^th^ week after operation) prior to the appearance of heart failure in aged rats (the 9^th^ week after operation). During the 2–7^th^ week after operation, no significant difference was observed in the alveolar space, lung interstice or peri-alveolar blood vessels in the BRL group, non-BRL group or Sham group. However, from the 5^th^ to the 7^th^ week after operation, the peri-alveolar blood vessels in the BRL group reveal slight dilation and blood stasis. Subsequently, during the 7–11^th^ weeks after operation, lung lesions in the non-BRL group were gradually characterized by interstitial edema, acinar cell vacuolization, and infiltration of inflammatory and congestion edema (Figure 2).

**Figure 2:** Lung histopathology at different times and in different groups. The lung tissues were observed with a Brightfield microscope under 40× magnification (Olympus BX 51, Japan). During the 2–5^th^ week after operation, no significant difference in alveolar space, lung interstice and peri-alveolar blood vessels from BRL group, non-BRL group or Sham group was observed. However, during the 5–7^th^ week after operation, the peri-alveolar blood vessels in the BRL group revealed slight dilation and blood stasis, and then during the 7–11^th^ week after operation, the lung lesions was gradually characterized by interstitial edema, acinar cell vacuolization, and infiltration of inflammatory and congestion edema in the BRL group. BRL group: HF group with β_3_-AR agonist BRL37344 injection; non-BRL: HF group without BRL37344 injection.

The article "Relationship between the Autoantibody and Expression of β3-Adrenoceptor in Lung and Heart" was retracted in 2025. Reasons: errors in the images; duplicated images; overlap with earlier publications; unreliable results or conclusions.

### Cardiac Histopathology in Aged Rats with Heart Failure

No nuclear degeneration was observed in the intercellular spaces in any of the 3 groups during the 2–7^th^ weeks after operation, however, during the 9–11^th^ week after operation, cardiac lesions in the BRL and non-BRL groups were gradually characterized by interstitial fibrosis, edema, degeneration, necrosis, and myocyte hypertrophy. It is notable that the cardiac lesions in the BRL group were more pronounced than those observed in the non-BRL group (Figure 3).

**Figure 3:** Cardiac histopathology at different times and in different groups. Representative images of myocardial cells at the 5^th^, 7^th^, 9^th^, and 11^th^ week [observed with a Brightfield microscope under 40× magnification (Olympus BX 51, Japan) were presented. During the 5–7^th^ week after operation, the myocardial cells revealed an ordered arrangement and normal intercellular space without nuclear degeneration. However, at the 9^th^ week, the time-dependent increase of interstitial fibrosis, edema, degeneration, necrosis, and myocyte hypertrophy was observed in the BRL group when compared to the Banded group. BRL group: HF group with β_3_-AR agonist BRL37344 injection; non-BRL: HF group without BRL37344 injection.

### The Expression of β_3_-AR MRNA and Protein in Lung and Heart

In the present study, we first demonstrated the polarity of the expression of β_3_-AR mRNA and protein in the lung and cardiac tissues from rats with heart failure. The expression levels of β_3_-AR mRNA and protein in lungs from the non-BRL group exhibited a negative correlation with the severity of heart failure (*p*<0.001) (Figure 4).

**Figure 4:** Expression of β3-AR mRNA by RT-PCR and β3-AR protein by Western blot in lung. (A) Representative analysis of β3-AR mRNA level by RT-PCR. Lane M: marker; bp: base pair; lane n5: the 5^th^ week, non-BRL group; lane n7: the 7^th^ week, non-BRL group; lane n9: the 9^th^ week, non-BRL group; lane n11: the 11^th^ week, non-BRL group. (B) Bar plot showed the data from all animals in the non-BRL group. Data were analyzed by ANOVA. β3-AR revealed a decrease with the deterioration of heart failure. (*p<0.05, versus non-BRL group 2 weeks prior to treatment). (C) Immunoblot of β3-AR protein in representative animals. Lane n5: the 5^th^ week, non-BRL group; lane n7: the 7^th^ week, non-BRL group; lane n9: the 9^th^ week, non-BRL group; lane n11: the 11^th^ week, non-BRL group. GAPDH: glyceraldehyde phosphate dehydrogenase. (D) Bar plot showed the data from all animals in each group. The data are analyzed by ANOVA. β3-AR protein revealed a decrease with the deterioration of heart failure. (*p<0.05, versus non-BRL group 2 weeks prior to treatment). BRL group: HF group with β_3_-AR agonist BRL37344 injection; non-BRL: HF group without BRL37344 injection.

The article "Relationship between the Autoantibody and Expression of β3-Adrenoceptor in Lung and Heart" was retracted in 2025. Reasons: errors in the images; duplicated images; overlap with earlier publications; unreliable results or conclusions.

Conversely, the expression levels of cardiac β_3_-AR mRNA and protein in both BRL and non-BRL groups exhibited a positive correlation with the severity of heart failure (*p*<0.001). More importantly, compared with the non-BRL group, the BRL group revealed a more obviously positive correlation with the severity of heart failure (*p*<0.01). These results suggested that β_3_-AR agonist might further activate the expression of β_3_-AR mRNA and protein in heart of the aged rats with heart failure (Figure 5).

**Figure 5:** Myocardiac β3-AR mRNA by RT-PCR and β3-AR Protein by Western blot. (A) Representative analysis of myocardiac β3-AR mRNA level by RT-PCR. Lane M: marker; bp: base pair; lane n5: the 5^th^ week, non-BRL group; lane n7: the 7^th^ week, non-BRL group; lane n9: the 9^th^ week, non-BRL group; lane n11: the 11^th^ week, non-BRL group; lane B5: the 5^th^ week, BRL group; lane B7: the 7^th^ week, BRL group; lane B9: the 9^th^ week, BRL group; lane B11: the 11^th^ week, BRL group. (B) Bar plot showed the data from myocardial tissues of all animals in each group. Data were analyzed by ANOVA. The expression of β3-AR was significantly higher at the 9^th^ and 11^th^ week in the BRL group than that in the Banded group (*p<0.05, BRL group vs. Banded group). The β3-AR revealed a time-dependent increase in each group (*p*<0.01). (C) Immunoblot of myocardiac β3-AR protein in representative animals. Lane n5: the 5^th^ week, non-BRL group; lane n7: the 7^th^ week, non-BRL group; lane n9: the 9^th^ week, non-BRL group; lane n11: the 11^th^ week, non-BRL group; lane B5: the 5^th^ week, BRL group; lane B7: the 7^th^ week, BRL group; lane B9: the 9^th^ week, BRL group; lane B11: the 11^th^ week, BRL group. GAPDH: glyceraldehyde phosphate dehydrogenase. (D) Bar plot showed the data from myocardiac tissues of all animals in each group. The data were analyzed by ANOVA. At each time point (except 5 wk), the expression of β3-AR protein was significantly higher in the BRL group than that in the Banded group. The expression of β3-AR protein revealed a time-dependent increase, and its expression at the 11^th^ week was significantly higher than that at the 5^th^ week (*p*<0.01, Banded group: 0.62±0.08 vs. 0.51±0.03; BRL group: 1.01±0.10 vs. 0.52±0.02). (**p<0.01, BRL group vs. Banded group). BRL group: HF group with β_3_-AR agonist BRL37344 injection; non-BRL: HF group without BRL37344 injection.

The article "Relationship between the Autoantibody and Expression of β3-Adrenoceptor in Lung and Heart" was retracted in 2025. Reasons: errors in the images; duplicated images; overlap with earlier publications; unreliable results or conclusions.

## Discussion

Three subtypes of β-receptors are expressed in normal hearts at various levels. The expression levels of β_1_-AR and β_2_-AR subtypes are approximately 70–80% and 20–30%, respectively, but β_3_-AR subtype can not be detected under normal conditions [18]. The β_3_-AR subtype is first characterized in human endomyocardial biopsies from transplanted hearts [7]. Moreover, different subtypes of β-receptors have different impacts on myocardial contractility. The myocardial contractility is increased by activated β_1_-AR and β_2_-AR subtypes but decreased by activated β_3_-AR subtype [19]. In senescent heart, both β_1_-AR and β_2_-AR subtypes are down-regulated [20], [21], but the up-regulation of β_3_-AR is reported by Birenbaum et al. [21], and it is never reported previously. In the present study, we have first demonstrated that the ascending aorta banding-induced heart failure in aged rats is an accurate and reliable model, but with a mortality up to 50%. In addition, our results suggest that the β_3_-AR agonist may be associated with the increased risk of death in aged rats with heart failure. Third, the frequencies and mean titer of anti-β_3_-AR autoantibody in aged patients and rats with heart failure are significantly higher than those within the control groups, and reveal an increase with diminishing heart function. Finally, the expression of lung β_3_-AR mRNA and protein could exhibit a negative correlation with the severity of heart failure, and is observed earlier than expression in the heart in the experiment. Conversely, the expression of β_3_-AR in cardiac tissues exhibits a positive correlation, which is further increased by the presence of β_3_-AR agonist. It is also notable that the serum levels of anti-β_3_-AR autoantibody are negatively correlated with the expression of lung β_3_-AR, but positively correlated with the expression of heart β_3_-AR. These results suggest that the plasma levels of anti-β_3_-AR autoantibody may act as a clinical reference index of prognosis in patients with heart failure, and may indirectly reflect the expression of β_3_-AR mRNA and protein in both lungs and heart. These findings suggest that the β_3_-AR and anti-β_3_-AR autoantibody play an important role in the senescent heart with heart failure. But we think it is the first step to reveal the link between the activation of β_3_-AR and the aggravated heart failure in the senescent heart. Further studies are needed to reveal the underlying mechanism. Birenbaum and colleagues have reported that the up-regulation of β_3_-AR plays an important role in the altered contractile response of β-adrenergic stimulation *via* induction of NOS1-nitric oxide in rat senescent heart [21]. But Gauthier has also reported that the negative inotropic effectinduced by β_3_-AR is obviously coupled to an activation of G_i/o_ proteins and the stimulation of the nitric oxide (NO) pathway in ventricular endomyocardial biopsy samples of heart transplant recipients. The NO production leads to an activation of soluble guanylyl cyclase leading to an increase in intracellular cGMP [11]. And the hypothesis of G_i/α_ inhibition of adenylate cyclase is theoretically considered because part of the negative inotropic effect of β_3_-AR agonists is insensitive to NOS inhibition. Therefore, β_3_-AR might activate growth or metabolic signaling(e.g. through activation of MAP kinases). Thus, future works should be performed to demonstrate these mechanisms in more models.

The article "Relationship between the Autoantibody and Expression of β3-Adrenoceptor in Lung and Heart" was retracted in 2025. Reasons: errors in the images; duplicated images; overlap with earlier publications; unreliable results or conclusions.

### Mortality Rate and Heart Failure in Aged Rats

The model of ascending aorta banding-induced chronic heart failure has been widely used to produce a time-dependent impairment of cardiac function [19], [22]. However, the model has not been previously applied using aged rats. The results of the current study indicate that ascending aorta banding-induced heart failure in aged rats is an accurate and reliable model, but with a mortality rate exceeding 50%. These early deaths appear to be due to anesthesia intolerance or acute heart failure. The mortality rate in BRL group is significantly higher than that in non-BRL group, suggesting that β_3_-AR agonist (BRL-37344) may further increase mortality rate in aged rats with heart failure.

On the other hand, we have used male rats in the experiment because estrogen plays a cardioprotective role in female rat hearts. The effects of estrogen during ischaemia-reperfusion injury are associated with the decreased cardiomyocyte contraction and expression of β_1_-AR, and increased expression of β_2_-AR [23].

### Anti-β_3_-AR Autoantibody and Heart Failure

In recent years, several studies have reported that the positive rates of anti-β_3_-AR autoantibody in patients with heart failure are remarkably higher than those in the control group [20], [24]. The results of our study demonstrate for the first time that, in aged patients with heart failure, the positive rate is associated with a 3- to 4-fold increase in anti-β_3_-AR autoantibody when compared with the normal control. Similarly, the positive rate in aged rats is positively correlated with the severity of heart failure. These results strongly suggest that the plasma level of anti-β_3_-AR autoantibody can act as a clinical reference index of the prognosis in patients with heart failure, especially aged patients.

### The Expression of Pulmonary β_3_-AR in Heart Failure

One of the most important findings from the present study is that the expressions of lung β_3_-AR mRNA and protein reveal gradual decrease in aged rats with heart failure, exhibiting a negative correlation with the severity of heart failure. Additionally, β_3_-AR agonist (BRL 37344) can further inhibit the expression of β_3_-AR mRNA and protein in pulmonary tissues. Moreover, it has been reported that β_3_-AR agonist can increase alveolar fluid clearance during lung injury and accelerate the amelioration of pulmonary edema. We therefore speculate that, with the anti-β_3_-AR autoantibody, similar to a β_3_-AR agonist, these protective effects may greatly decrease or even disappear with gradually decreasing β_3_-AR expression in pulmonary tissues. Furthermore, β_3_-AR reveals a significant decrease in density and activity, thus resulting in a significant pulmonary congestion or edema.

The article "Relationship between the Autoantibody and Expression of β3-Adrenoceptor in Lung and Heart" was retracted in 2025. Reasons: errors in the images; duplicated images; overlap with earlier publications; unreliable results or conclusions.

### Cardiac β_3_-AR Expression in Heart Failure

Multiple studies have established that in normal heart tissues, the negative inotropic effect induced by β_3_-AR may play a safety role during intense adrenergic stimulation such as stress and strong physical effort. Thus, over-expression of β_3_-AR may protect against cardiac damage induced by the high catecholamine level present in heart failure, particularly during the early stages. However, during the worst stages of heart failure, the down-regulation of cardiac β_1_-AR and β_2_-AR, and concomitant decrease in adenylyl cyclase activity result in a significant enhancement of cAMP-mediated negative inotropic effects, thereby enhancing myocardial depression [8], [10], [25]. Interestingly, β_3_-AR expression is up-regulated 2–3 times faster in the failing heart when compared with the non-failing heart [26]. The negative inotropic effect of the β_3_-AR agonist may therefore exacerbate cardiac dysfunction and profoundly aggravate systolic and diastolic dysfunction.

### The Relationship between β_3_-AR and Anti-β_3_-AR Autoantibodies

In our aged rat model, increasing impairment of heart function is associated with a 3- to 4-fold increase in β_3_-AR expression in the heart. At the same time, the serum level of anti-β_3_-AR autoantibodies is associated with a 3- to 4-fold increase. Contrary to the results observed in the heart, a gradual decrease in the expression of β_3_-AR in the lung is observed. These data suggest that in the case of lung, the anti-β_3_-AR autoantibody, as β_3_-AR agonists, can increase continuous negative inotropic effects that can further inhibit the heart function, and at the same time, due to the significant increase in the expression of pulmonary β_3_-AR, the action of alveolar fluid clearance may be inhibited, resulting in increasingly impaired heart function. We therefore conclude that the serum level of anti-β_3_-AR autoantibody can act as a reference index of the prognosis in aged patients with heart failure, and indirectly reflect the expression of β_3_-AR mRNA and protein in the lungs and heart at different stages.

The article "Relationship between the Autoantibody and Expression of β3-Adrenoceptor in Lung and Heart" was retracted in 2025. Reasons: errors in the images; duplicated images; overlap with earlier publications; unreliable results or conclusions.

### Conclusion

The ascending aorta banding-induced heart failure model in aged rats is an accurate and reliable model, but is associated with high mortality rate. During the development of heart failure, pathological changes of lung injury preceded myocardial injury. The expression of β_3_-AR mRNA and protein in pulmonary tissues reveals a gradual decrease, but the expression in myocardial tissues reveals an increase and can further be promoted by β_3_-AR agonist. The anti-β_3_-AR autoantibodies can increase gradually as the progression of heart failure. The serum levels of anti-β_3_-AR autoantibody may then act as a reference index, indirectly reflecting the expression of β_3_-AR mRNA and protein in lungs and heart at different stages.

## Materials and Methods

### Ethics Statement

The present human study complied with the Declaration of Helsinki and was approved by the Ethics Committee and the Prescription and Therapeutic Committee (10-S-6) of Capital Medical University Beijing Chao-yang Hospital. All subjects provided written informed consented prior to admission into the study.

All animal experiments were approved by the Institutional Animal Care and Use Committee of Capital Medical University (10-A-35). All surgeries were performed under isoflurane/oxygen anesthesia and all efforts were made to minimize suffering including the use of buprenorphine for pain management after surgery.

### Study Cases

Outpatients from Beijing Chao-yang Hospital of China were the source of the samples collected for the determination the anti-β_3_-AR autoantibody. Sixty-nine heart failure patients were selected for this study. Criteria for patient selection included: aged 65 years or older defined according to New York Heart Association (NYHA) functional classes II-IV; less than 45% left ventricular ejection fractions on echocardiograms; no apparent severe hepatic and renal dysfunction; no previous medication of ACEI, diuretic and/or digoxin. The normal control groups (NC) were comprised of 27 healthy individuals exhibiting normal clinical, ECG and echocardiography examinations, and matched ages and sexes with the heart failure patients.

### Animal Models and Drug Administration

Healthy 20 month-old male Wistar rats, weighing 500 to 550 g, were selected for this study. Animals were classified randomly into 2 experimental groups and a control group. Experimental animals (n = 140) were subjected to aorta banding, in which the ascending aorta was banded (steel wire area/ascending aorta area = 75%) according to the methods of Brown, et al [22]. In the sham-operated control group (n = 35), the animals were treated with the same surgical procedures, but without the aortic banding. After 5 weeks, aged Wistar rats from the aorta-banding group were divided into a BRL group (n = 50) and a non-BRL group (n = 40). The BRL group received β_3_-AR-selective agonist (BRL37344 (4-[2-[(2-(3-chlorophenyl)-2-hydroxyethyl) amino] propyl] phenoxyacetic acid) (Sigma-Aldrich Co. USA) at a dose of 0.4 nmol·kg^−1^·min^−1^ via a vena caudal injection sustained for 10 minutes, twice weekly for 6 weeks, while an equivalent dose of normal saline was administrated in the non-BRL group.

The article "Relationship between the Autoantibody and Expression of β3-Adrenoceptor in Lung and Heart" was retracted in 2025. Reasons: errors in the images; duplicated images; overlap with earlier publications; unreliable results or conclusions.

### Hemodynamic Measurement and LVW/BW

Eight animals were anesthetized with urethane (20%, 1 g/kg). A cannula connected to a pressure transducer was inserted along the carotid artery into the left ventricle to measure the following primary and derived variables: heart rate, left ventricle end-systolic pressure, left ventricle end-diastolic pressure and the maximal rate of rise and decline in left ventricle pressure (dP/dt_max_ and dP/dt_min_) by opened thorax. All pressures were measured with a pressure transducer connected to a polygraph recorder (BL-420F, Chengdu Taimeng Technology Co., LTD, China), stored, and displayed on a personal computer. The lung and heart tissues were rapidly excised and frozen in liquid nitrogen, and then stored at −80°C until use.

The bodies and the left ventricles of each rat were weighed, and the ratio of left ventricular weight to body weight (LVW/BW) was calculated.

### Microscopic Structure Inspection of Lung and Heart

The lung and heart were filled with 10% formalin for fixation, and coated in gauze for histopathological examination. All tissue specimens were cut into 5-mm-thick cross-sections, fixed in 10% formalin, dehydrated, and embedded in paraffin. Slices with 5 µm in thickness were obtained from the sections and stained with hematoxylin-eosin. The tissues were observed with a Brightfield microscope under 40× magnifications (Olympus BX 51, Japan).

### Serum Sampling and Anti-β_3_-AR Determination

Two milliliters of blood were withdrawn from the antecubital vein in patients with heart failure and in the control cases. Throughout the experiment of aged rats, 2 mL of blood samples were taken from the carotid arteries of subjects from all groups. Samples were collected before treatment, and at the 5^th^, 6^th^,7^th^, 8^th^,9^th^, 10^th^ and 11^th^ week after treatment. The sera were separated by centrifugation (3000 rpm, Beckman CS-5R Centrifuge) for 10 min and stored at −80°C until needed for assay.

The article "Relationship between the Autoantibody and Expression of β3-Adrenoceptor in Lung and Heart" was retracted in 2025. Reasons: errors in the images; duplicated images; overlap with earlier publications; unreliable results or conclusions.

The peptides with terminal cysteines corresponding to the sequence of the second extracellular loop of the human β_3_-AR (residues176–202: Q-W-W-R-V-G-A-D-A-E-A-Q-R-C-H-S-N-P-R-C-C-A-F-A-S-N-M-C) were synthesized by the Biological Institute of CAMS &PUMC, Beijing, using the solid phase method of Merrifield. The purity of these peptides was evaluated by HPLC on a Vydac C−18 column and by amino acid analysis on an automated amino acid analyzer (Beckman instruments, Inc, Palo Alto, CA, USA). The peptides in rats were nearly identical, except for residues shaded in the following sequence of β_3_-AR (residues173–199:Q-W-W-R-V-G-A-D-A-E-A-Q-E-C-H-S-N-P-R-C-C-S-F-A-S-N-M-C).

Anti-β_3_-AR autoantibody was determined by enzyme-linked immunosorbent assays (ELISA). Both the study population and rats were defined as being positive or negative based on the presence or absence of anti-β_3_-AR autoantibody. The ELISA protocol as described by Fu, et al. was used to screen for the presence of autoantibodies [1], [2], [3], [4].

### RT-PCR and the Expression of β_3_-AR

Amplification of β_3_-AR by PCR was completed in a 50-µL reaction mixture containing 100 mM Tris-HCl (pH 8.3), 500 mM KCl, 15 mM MgCl_2_, 200 µM dNTPs, 20 pmol each of the primers, 1 unit of Taq polymerase, and 2 µL of DNA template. Amplification was performed with a thermal cycler (PTC-200 Peltier, Bio-RAD) using the following parameters: initial denaturation at 95°C for 3 min; denaturation at 94°C for 30 s, annealing at 54°C for 30 s, and extension at 72°C for 90 s for 40 cycles; and a final extension at 72°C for 10 min. For the β-actin reaction, a 50-µL reaction mixture containing 100 mM Tris-HCl (pH 8.3), 500 mM KCl, 200 µM dNTPs, 20 pmol each of the primers, 15 mM MgCl_2_ and 1 unit of Taq polymerase, was used. The conditions for the reaction were as follows: initial denaturation at 95°C for 3 min; 35 cycles of denaturation at 94°C for 30 s, annealing at 51°C for 30 s, and extension at 72°C for 90 s; and a final extension at 72°C for 10 min. PCR products were separated using 1% agarose gel and visualized on a gel documentation system (Vilber Lourmat Co., France) after staining with ethidium bromide.

### Western Blot and Expression Level of β_3_-AR Protein

Lung and cardiac tissues were homogenized in ice-cold homogenization buffer. Total protein was isolated from tissues and the concentration was determined using the Bradford method. Crude protein extracts (80 µg) were separated on a 10% SDS-polyacrylamide gel and then transferred to nitrocellulose membranes. The membranes were blocked for 1 h at room temperature in TBS-T containing 5% non-fat milk, and probed with primary antibodies against GAPDH and β_3_-AR (Santa Cruz Biotechnology, USA). The primary antibodies were diluted in TBS-T (1:1,000). Either alkaline phosphatase conjugated goat anti-mouse (GAPDH) or goat anti-rabbit (β_3_-AR) antibody was diluted to 1:3,000 in TBS-T and used as a secondary antibody with 1 h incubation. The bands on the blots were visualized using western blue (Promega, USA) and were semi-quantified using a computer image analysis system. The expression level of β_3_-AR protein was normalized to GAPDH.

The article "Relationship between the Autoantibody and Expression of β3-Adrenoceptor in Lung and Heart" was retracted in 2025. Reasons: errors in the images; duplicated images; overlap with earlier publications; unreliable results or conclusions.

### Data Analysis

All data, with the exception of antibody titers, are expressed as mean value ± SEM. Antibody titers reported as geometric means and differences between data sets were evaluated by unpaired Student’s *t-*test. All other data were evaluated by analysis of variance. In all cases, a statistically significant difference was considered at *p*<0.05. An anti-β_3_-AR positive score were defined as a ratio [(sample OD - blank OD)/(negative contrast OD - blank OD)] of ≥2.1. Analyses were performed with the GraphPad Prism 4.0 software package (San Diego, CA).

## References

[1] FuML, HoebekeJ, MatsuiS, MatobaM, MagnussonY, et al (1994) Autoantibodies against cardiac G-protein-coupled receptors define different populations with cardiomyopathies but not with hypertension. Clin Immunol Immunopathol 72: 15–20.802018810.1006/clin.1994.1101

[2] ZhangL, HuD, LiJ, WuY, LiuX, et al (2002) Autoantibodies against the myocardial beta1-adrenergic and M2-muscarinic receptors in patients with congestive heart failure. Chin Med J (Engl) 115: 1127–1131.12215275

[3] DandelM, WallukatG, PotapovE, HetzerR (2012) Role of beta(1)-adrenoceptor autoantibodies in the pathogenesis of dilated cardiomyopathy. Immunobiology 217: 511–520.2182075510.1016/j.imbio.2011.07.012

[4] HaberlandA, WallukatG, DahmenC, KageA, SchimkeI (2011) Aptamer neutralization of beta1-adrenoceptor autoantibodies isolated from patients with cardiomyopathies. Circ Res 109: 986–992.2186869610.1161/CIRCRESAHA.111.253849

[5] HerdaLR, FelixSB, BoegeF (2012) Drug-like actions of autoantibodies against receptors of the autonomous nervous system and their impact on human heart function. Br J Pharmacol 166: 847–857.2222062610.1111/j.1476-5381.2012.01828.xPMC3412294

[6] DuY, YanL, DuH, WangL, DingF, et al (2012) beta1 -adrenergic receptor autoantibodies from heart failure patients enhanced TNF-alpha secretion in RAW264.7 macrophages in a largely PKA-dependent fashion. J Cell Biochem 113: 3218–4228.2262817410.1002/jcb.24198

[7] GauthierC, TavernierG, CharpentierF, LanginD, LeMH (1996) Functional beta3-adrenoceptor in the human heart. J Clin Invest 98: 556–562.875566810.1172/JCI118823PMC507461

The article "Relationship between the Autoantibody and Expression of β3-Adrenoceptor in Lung and Heart" was retracted in 2025. Reasons: errors in the images; duplicated images; overlap with earlier publications; unreliable results or conclusions.

[8] RozecB, GauthierC (2006) beta3-adrenoceptors in the cardiovascular system: putative roles in human pathologies. Pharmacol Ther 111: 652–673.1648077110.1016/j.pharmthera.2005.12.002

[9] ZhaoQ, WuTG, JiangZF, ChenGW, LinY, et al (2007) Effect of beta-blockers on beta3-adrenoceptor expression in chronic heart failure. Cardiovasc Drugs Ther 21: 85–90.1744082410.1007/s10557-007-6016-4

[10] RasmussenHH, FigtreeGA, KrumH, BundgaardH (2009) The use of beta3-adrenergic receptor agonists in the treatment of heart failure. Curr Opin Investig Drugs 10: 955–962.19705338

[11] GauthierC, LeblaisV, KobzikL, TrochuJN, KhandoudiN, et al (1998) The negative inotropic effect of beta3-adrenoceptor stimulation is mediated by activation of a nitric oxide synthase pathway in human ventricle. J Clin Invest 102: 1377–1384.976933010.1172/JCI2191PMC508985

[12] GermackR, DickensonJM (2006) Induction of beta3-adrenergic receptor functional expression following chronic stimulation with noradrenaline in neonatal rat cardiomyocytes. J Pharmacol Exp Ther 316: 392–402.1618370810.1124/jpet.105.090597

[13] BossardF, SilantieffE, Lavazais-BlancouE, RobayA, SaganC, et al (2011) beta1, beta2, and beta3 adrenoceptors and Na+/H+ exchanger regulatory factor 1 expression in human bronchi and their modifications in cystic fibrosis. Am J Respir Cell Mol Biol 44: 91–98.2020329210.1165/rcmb.2009-0372OC

[14] NgTM, MungerMA, LombardiWL, DoingTH, RyujinDT, et al (2002) Chronically inhaled salmeterol improves pulmonary function in heart failure. J Cardiovasc Pharmacol 40: 140–145.1207258710.1097/00005344-200207000-00017

[15] MaronMB, LutherDJ, PilatiCF, OhanyanV, LiT, et al (2009) Beta-adrenoceptor stimulation of alveolar fluid clearance is increased in rats with heart failure. Am J Physiol Lung Cell Mol Physiol 297: L487–495.1959245710.1152/ajplung.90629.2008

[16] EvansBA, PapaioannouM, BonazziVR, SummersRJ (1996) Expression of beta 3-adrenoceptor mRNA in rat tissues. Br J Pharmacol 117: 210–216.882536510.1111/j.1476-5381.1996.tb15176.xPMC1909365

[17] LiNJ, LiW, HeP, GuX, LiSQ (2010) Effect of beta3-adrenergic agonists on alveolar fluid clearance in hypoxic rat lungs. Chin Med J (Engl) 123: 1028–1033.20497709

[18] StrosbergAD (1997) Structure and function of the beta 3-adrenergic receptor. Annu Rev Pharmacol Toxicol 37: 421–450.913126010.1146/annurev.pharmtox.37.1.421

[19] GauthierC, Seze-GoismierC, RozecB (2007) Beta 3-adrenoceptors in the cardiovascular system. Clin Hemorheol Microcirc 37: 193–204.17641409

[20] XiaoRP, TomhaveED, WangDJ, JiX, BoluytMO, et al (1998) Age-associated reductions in cardiac beta1- and beta2-adrenergic responses without changes in inhibitory G proteins or receptor kinases. J Clin Invest 101: 1273–1282.950276810.1172/JCI1335PMC508681

The article "Relationship between the Autoantibody and Expression of β3-Adrenoceptor in Lung and Heart" was retracted in 2025. Reasons: errors in the images; duplicated images; overlap with earlier publications; unreliable results or conclusions.

[21] BirenbaumA, TesseA, LoyerX, MicheletP, AndriantsitohainaR, et al (2008) Involvement of beta 3-adrenoceptor in altered beta-adrenergic response in senescent heart: role of nitric oxide synthase 1-derived nitric oxide. Anesthesiology 109: 1045–1053.1903410110.1097/ALN.0b013e31818d7e5a

[22] BrownRH, WaltersDM, GreenbergRS, MitznerW (1999) A method of endotracheal intubation and pulmonary functional assessment for repeated studies in mice. J Appl Physiol 87: 2362–2365.1060119010.1152/jappl.1999.87.6.2362

[23] WuQ, ZhaoZ, SunH, HaoYL, YanCD, et al (2008) Oestrogen changed cardiomyocyte contraction and beta-adrenoceptor expression in rat hearts subjected to ischaemia-reperfusion. Exp Physiol 93: 1034–1043.1846906810.1113/expphysiol.2007.041939

[24] LiMX, WangXL, TangJN, LiuXJ, TianJ, et al (2005) [Distribution and property of anti-beta3-adrenoceptor autoantibody in patients with heart failure]. Zhonghua Xin Xue Guan Bing Za Zhi 33: 1114–1118.16563283

[25] ZhangZS, ChengHJ, OnishiK, OhteN, WannenburgT, et al (2005) Enhanced inhibition of L-type Ca2+ current by beta3-adrenergic stimulation in failing rat heart. J Pharmacol Exp Ther 315: 1203–1211.1613570210.1124/jpet.105.089672

[26] MoniotteS, KobzikL, FeronO, TrochuJN, GauthierC, et al (2001) Upregulation of beta(3)-adrenoceptors and altered contractile response to inotropic amines in human failing myocardium. Circulation 103: 1649–1655.1127399210.1161/01.cir.103.12.1649

